# Biostatistics of VHL-Gene Transfection in the Health Informatics Analysis of Renal Cell Carcinoma

**DOI:** 10.1155/2022/5297580

**Published:** 2022-01-07

**Authors:** Yunxiang Gong, Degang Wang, Wengang Wang

**Affiliations:** Department of Urology Surgery, Fuxin Centre Hospital, Fuxin 123000, China

## Abstract

**Objective:**

In this paper, we study the role of the VHL gene in regulating the proliferation and apoptosis of renal cell carcinoma, as well as the safety and transfection efficiency of ultrasound microbubble gene transfection technology.

**Method:**

We use kidney cancer cell lines as an in vitro research object and apply ultrasound microbubble gene transfection technology to transfect the VHL gene into kidney cancer cell line (786-0). The proliferation and apoptosis of cells were measured to clarify the inhibitory effect of the VHL gene in renal cell carcinoma. After that, pEGFP-VHL was transfected using ultrasonic microbubble and liposome gene transfection techniques, respectively, and the transfection efficiency was measured by immunofluorescence.

**Results:**

Compared with untreated and 786-0 cells that are transfected with empty vector, the expression level of VHL gene mRNA in 786-0 cells that are transfected with pcDNA3.1-VHL was significantly increased, and the cell growth inhibition rate was significantly higher. The rate of apoptosis increased significantly. Transfection efficiency of the pEGFP-VHL gene after transfection of 786-0 cells for 48 h: control group 0, liposome group (35.55 ± 2.77) %, ultrasound microbubble group (18.27 ± 2.83) %, and two transfection methods on cells. There is no significant difference in the impact of vitality.

**Conclusion:**

VHL gene expression can significantly inhibit the proliferation ability of renal cancer cell line 786-0 and promote its apoptosis. VHL gene is a potential target for gene therapy of kidney cancer.

## 1. Background

Renal cell carcinoma that is abbreviated as RCC, referred to as kidney cancer, accounts for 2-3% of all adult malignant tumors. Renal cancer deaths worldwide are more than 100,000 cases per year [1]. The incidence of kidney cancer involves multiple genes, of which the Von Hippel-Lindau (VHL) gene is most closely related to kidney cancer. VHL gene has the functions of regulating transcription, regulating cell cycle, and stabilizing cell growth-related genes.

The VHL gene suppresses the formation of the transcription elongation factor Elongin complex through pVHL and regulates the expression of cell growth-related genes. pVHL is also related to cell proliferation, apoptosis, and tumor infiltration and metastasis. VHL gene mutation, deletion, and hypermethylation are closely related to the occurrence of renal cell carcinoma. Research has found [2] that the VHL gene-hypoxia-inducible factor-hypoxia response gene pathway (VHL-HIF-HRG pathway) plays an important role in kidney cancer.

VHL disease involves multiple systemic lesions, including kidney cancer, hemangioblastoma, pheochromocytoma, pancreas, and epididymal cyst. Among them, the incidence of kidney cancer is as high as 28-45%. Lalif [3] successfully cloned the VHL gene in 1993 and confirmed that the root cause of VHL disease is VHL gene inactivation, and VHL exists in more than 98% of VHL diseases. The gene is inactivated. The total length is about 15 kb and encodes 4.7 kb long mRNA. The protein product produced by the VHL gene encoding is called protein VHL (pVHL).

The molecular weight of the VHL protein is 28 -30 KD, including 213 amino acids, called p30 or pVHLL protein; the VHL gene can also encode a protein with a molecular weight of 19 KD, called pl9 or pVHLS protein. The pl9 protein has a similar function to the p30 protein. It is an isomer that is transcribed at the second transcription start site of the VHL gene. It is not clear why pl9 protein is produced. pVHL30 and pVHL 19 have different localizations in cells, and their functions have not yet been fully clarified. VHL19 is mainly located in the nucleus, which has a higher affinity for the nucleus than pVHL30. In the cytoplasm, pVHL30 is connected by tiny tubes, allowing mRNA to be specifically expressed in tissues. The homologous VHL has also been identified in mice, worms, and fruit flies [4].

The main biological feature of kidney cancer is the abundance of blood vessels. Angiogenesis requires four steps: degradation of extracellular matrix, migration of vascular endothelial cells, proliferation of endothelial cells, and vascular shaping. The process of angiogenesis requires the participation of a series of cytokines. These factors are called angiogenic factors. Due to the abnormality of the VHL gene, the VHL-HIF-HRG signaling pathway is continuously activated, causing tumor cells to synthesize and secrete a large amount of angiogenic factors. VHL is closely related to the formation of renal tumor blood vessels. The VHL-HIF-HRG pathway provides new targets for the treatment of kidney cancer in multiple links [5]. At present, the molecular biological mechanism of kidney cancer is continuously deepened, and molecular targeted therapy must be paid more and more attention.

VHL-HIF-HRG pathway provides a new target for the treatment of kidney cancer in multiple links. Humans control the growth of tumors by blocking the expression of downstream target genes of HIF-a, such as VEGF, PDGF, and TGF-a. A variety of molecular-targeted therapeutic drugs have come out in succession [6]. However, these drugs target the downstream target genes in the VHL-HIF-HRG pathway, and the VHL gene is the starting point of the VHL-HIF-HRG pathway. The VHL gene itself can be used as a target gene for gene therapy. Taking VHL as a target, transfecting it into renal cancer cells with appropriate methods, increasing the expression of the VHL gene, and correcting the apoptosis defects of tumor cells are very important treatment strategies.

Renal cancer cells lacking the VHL gene can form normal-sized tumors in nude mice, and the tumors formed after the introduction of wild-type VHL genes become significantly smaller, and even do not form tumors. Jacob et al. [7] reported that the introduction of VHL gene into arterial endothelial cells through adenovirus can effectively inhibit the proliferation of endothelial cells. However, how to transfer the VHL gene safely, efficiently, specifically, and stably to tumor target cells for gene therapy is an urgent problem to be solved. In recent years, ultrasound has attracted much attention. Studies by scholars at home and abroad have shown that microbubble contrast agents can be promoted by ultrasound-mediated microbubble rupture method [8]. The safe and effective targeted transfer of the target gene may become a new method of gene therapy SI. Through the in-depth study of VHL gene and the development of gene transfection technology, gene therapy for kidney cancer with VHL gene as a target has bright prospects.

## 2. Methodology

### 2.1. Experimental Subjects

The human kidney cancer cell line 786-0 is universal, suitable for this experiment, and provides experimental objects for universal kidney cancer gene therapy.

### 2.2. Sources of pcDNA3.1(+), pcDNA3.1-VHL, and pEGFP-VHL

The eukaryotic expression vector pcDNA3.1(+) was from Beijing Promega Biotechnology Co., Ltd. Recombinant plasmid pcDNA3.1-VHL was constructed and identified by Tianjin Saier Biological Company. The pEGFP-VHL fusion gene expression vector was constructed and identified by Tianjin Saier Biological Company.

### 2.3. Experimental Cells

786-0 cells were trained in RPMI1640 medium consisting 100 g/ml penicillin >100 g/ml streptomycin and 10% fetal bovine serum in a 37°C, 5% CO_2_ incubator.

### 2.4. Cell Transfection

Cell transfection procedures are as follows.

(1) Experiment grouping and experiment preparation:
  - The experiment is categorized as (1) control group, (2) pcDNA3.1 (+) group, and (3) pcDNA3.1-VHL group
  - Transfection using ultrasonic microbubble gene transfection method
  - The parameters of the ultrasonic gene transfection therapy instrument are power 1.2 W, frequency 1000 Hz, and irradiation time 30 s. Ultrasonic microbubble concentration is 1 × 106/ml; after preparing ultrasonic microbubble contrast agent with sterile double distilled water, remember count the microbubble concentration and take out the required volume according to the desired final concentration
  - Preparation of the microbubble contrast agent/pcDNA3.1(+) mixture: mix pcDNA3.1(+) 10 g/well with SonoVue microbubble 100 g/well, let stand on ice for 20 minutes, and then it can be used for transfection
  - Preparation of cDNA3.1-VHL mixture of microbubble contrast agent: mix pcDNA3.1(+) 10 g/well with SonoVue microbubble 100 g/well, let stand on ice for 20 minutes, and then it can be used for transfection
(2) The 786-0 cells in good growth state were cultured the day before transfection, (0.5 − 2) × 105 cells/well, 2 ml per well without antibiotic medium, and cells per well when transfected the next day grows to 70-80%
(3) After washing the cells with PBS, we prepare a cell suspension without serum medium, 300 g/well, making the cell density 1 × 107 cells/ml
(4) Add the above mixture according to the requirements of each group, that is, pcDNA3.1(+) group plus microbubble contrast agent cDNA3.1(+) mixture, pcDNA3.1-VHL group plus microbubble contrast agent/pcDNA3.1-VHL mixture. Simultaneously give ultrasound irradiation under the above conditions. The control group only added serum-free medium. After continuing the culture for 6 hours, discard the old culture medium and add the normal culture medium at the same time and place it in a 37°C incubator to continue the culture

### 2.5. RT-PCR Analysis

#### 2.5.1. RNA Extraction

After 48 h after transfection, aspirate the culture medium in each group of culture flasks, add 1 ml Trizol to make them even without passing through the bottom of the culture flask, let stand for 5 min, and shake the culture flask around. Blow the cells repeatedly with a pipette and then move to a 1.5 ml Eppendorf tube. We included 200 *μ*l of chloroform, mix well by inversion, centrifuge at 14000 rpm, 4°C for 15 min. We aspirate supernatant into a new Eppendorf tube add 600 g of -20C precooled isopropanol to each tube. Centrifuge at l4000 rpm, 4 C for 10 min, discard the supernatant. Add 1 ml of 75% ethanol to each tube, pop up the pellet, centrifuge at 12000 rpm for 10 min, and discard the supernatant. Repeat step f-times. Leave to dry for 5 minutes at room temperature. Add 20 ml RNase-free water to each tube and dissolve for 5 min. After the precipitate is completely dissolved, remove 1 ml of each tube. The UV luminosity is A260 and A280 respectively.

#### 2.5.2. Using mRNA for RT-PCR Reaction

- Based on the genetic information of VHL, Primer Premier 5.0 software was used to design RT-PCR primers for VHL. The primer sequences are as follows:

VHL upstream primer: 5′-TACCGAGTGTATACTCTGAAAG-3′.

Downstream primer: 5′-GCTCCTGTGTCAGCCGCTCC-3′.

3-actin upstream primer: 5′-CGTGACATTAAGGAGAAGCTG-3′.

Downstream primer: 5′-CTAGAAGCATTTGCGGTGGAC-3.

(b) Take 5ug RNA and perform reverse transcription reaction using MMLV reverse transcriptase and related reagents

### 2.6. Flow Cytometry to Detect Apoptosis

48 h after transfection, we start the detection of apoptosis; aspirate the cell culture solution, wash the cells once with IxPBS solution, aspirate the PBS solution, add digestion solution (0.1% trypsin, 0.02% EDTA) 500 m, and act until the cell morphology changes. When the gap increases, we aspirate the digestion solution to stop digestion; we repeatedly blow the cells with Ixbinding buffer 200 and transfer cell suspension to a centrifuge tube; take 100 g of the cell suspension to a 1.5 ml centrifuge tube and add Annexin-VR-PE 10^1, after flicking and mixing, avoid light and ice bath for 20-30 min; we add Ixbinding buffer 380^1, then add 7-AAD 10 g, flick and mix; and finally, we detect it on flow cytometer.

### 2.7. MTT Detection Cell Value-Added Ability

We set up untreated group, pcDNA3.1 (+) group, and pcDNA3.1-VHL group, and each group has 3 complex wells. Digest the cells with 0.25% trypsin, centrifuge, inoculate 0.5 × 104 cells/well in a 96-well culture plate, 200 cell suspension per well, 3%, 5% CO_2_ incubator incubate overnight. When the degree of normal cell adhesion and fusion was 70~80%, the treatment group was subjected to the abovementioned ultrasound microbubble transfection conditions. After continuing to cultivate for 6 hours, discard the old culture medium and add the normal culture medium at the same time and place it in a 37°C incubator to continue the culture. Remove the culture plate, add MTT 5 mg/ml to each well, and place in 5% CO_2_ incubator for 4 hours.

We took away the culture plate, add 150^11 DMSO to each well to stop the reaction, shake for 10 min, and dissolve the purple crystals. The microplate reader measures the absorbance value (A570 value) of each well with a wavelength of 570 nm. Measure every 12 hours, record the result, and draw a curve.

### 2.8. Detection of Transfection Efficiency

There are the following categories: control group, pEGFP − VHL + liposome group, and PEGFP − VHL + ultrasound microbubble group. 786-0 cells were cultured in RPMI1640 with 100 g/m 1 penicillin, 100 g/ml streptomycin, and 10% fetal bovine serum in a 37°C, 5% CO2 incubator, whereby the cells used were all in the logarithmic growth phase. VHL cells in good growth state were cultured in 24-well plates and transfected when the cells grew to 70-80%. pEGFP − VHL + ultrasonic microbubble group: the pEGFP-VHL plasmid was transfected into 786-0 using the ultrasonic microbubble method. In the control group, only 1640 serum-free medium was added. After culturing for 48 hours, observe the transfection efficiency of the cells.

### 2.9. The Effect of Transfection

Our procedures are as follows:

1. A control group (medium and cells), a zero-adjusting group (medium), a liposome + pcDNA3.1 (+) group, an ultrasonic microbubble + pcDNA3.1 (+), and three complex wells in each group
2. Digest the cells with 0.25% trypsin, centrifuge, inoculate 0.5 × 104 cells/well in a 96-well culture plate, 200 g of cell suspension per well, and only add the equivalent in the zero-adjusting group amount of culture medium
3. When the normal growth and fusion degree of the adherent cells are 70% to 80%, the liposome + pcDNA3.1 (+) group and ultrasonic microbubbles + pcDNA3.1 (+) are transfected
4. Liposome + pcDNA3.1(+) group: the liposome can transfect pcDNA3.1(+) vector 786-0
5. Ultrasound microbubbles + pcDNA3.1(+) group: the pcDNA3.1(+) vector was transfected with 786-0 using the ultrasonic microbubbles method
6. Put the culture plate in 37°C, 5% CO_2_ incubator for 48 h, add 20 g of MTT to each well, continue culturing for 4 h, discard the supernatant, add 150 g DMSO to each well to stop the reaction, and shake for 10 min

### 2.10. Statistics

Data are statistically processed based on SPSS 12.0 software. Each analysis has at least three results. We used the mean ± standard deviation, using *t* test. *P* < 0.05 was considered to be significant and statistically significant.

## 3. Results

### 3.1. Semiquantitative Analysis of VHL Gene Expression

Results of RT-PCR analysis demonstrated that the relative IOD values of the mRNA levels of 786-0 cells untreated, transfected with pcDNA3.1(+) and transfected with pcDNA3.1-VHL, were 0.25 ± 0.03, 0.27 ± 0.05, and 0.73 ± 0.04, respectively. Compared with untreated and transfected 786-0 cells with pcDNA3.1(+), the expression level of VHL gene mRNA in 786-0 cells transfected with pcDNA3.1-VHL was significantly increased (*P* < 0.05): untreated and transfected. We note the similarity in expression level of VHL mRNA in 786-0 cells infected with pcDNA3.1 (+) (*P* > 0.05), as shown by Figure 1.

### 3.2. Flow Cytometry to Detect Apoptosis

The results of flow cytometry demonstrated that the apoptosis rates of 786-0 cells untreated, transfected with pcDNA3.1(+) and transfected with pcDNA3.1-VHL after 48 h of transfection, were 0.14%, 0.29%, and 22.74, respectively (Figures 2 and 3). Compared with untreated and transfected 786-0 cells with pcDNA3.1(+), the apoptosis rate of 786-0 cells transfected with pcDNA3.1-VHL was significantly increased. There are no significant difference in the apoptotic rate between untreated and 786-0 cells transfected with pcDNA3.1(+). It indicated that after transfection of VHL gene, the apoptosis rate of 786-0 cells increased.

Figure 3 shows that 48 hours after transfection, the apoptotic rate of each group was detected using a loss cytometer. FL1 (abscissa) is Annexin-VR-PE fluorescence signal value to detect phosphatidylserine; FL2 (ordinate) is 7-AAD fluorescence signal value to detect DNA. (1) Phosphatidylserine in the normal cell membrane is inside the membrane, and Annexin-V-R-PE cannot stain it; the cell membrane is intact, 7-AAD cannot be stained, and the corresponding points are distributed in the Q3 area. (2) The phosphatidylserine outside H, Annexin-VR-PE staining of the apoptotic cell membrane was positive; but the cell membrane was intact, 7-AAD could not be stained, and the corresponding points were distributed in the Q4 area. (3) Late apoptotic cells, necrotic cells, and other cell membranes of dead cells were broken, Annexin-VR-PE and 7-AAD could be stained, and the corresponding points were distributed in the Q2 area. The data were from at least three independent experiments. There was a difference at *P* < 0.05. Figure 3 demonstrated that 48 hours after transfection, the apoptosis rate of each group is from at least three independent experiments.

### 3.3. MTT to Detect Cell Growth

The proliferation curve (Figure 4) showed that there was no difference between untreated and transfected pcDNA3.1(+) 786-0 cell growth curves (*P* > 0.05), indicating that the cell proliferation characteristics after transfection with empty vector were not affected. The growth curve of 786-0 cells transfected with pcDNA3.1-VHL is below the two. There is a significant difference in cell proliferation ability between the pcDNA3.1-VHL group and the untreated group and the transfected pcDNA3.1(+) group (PV0.05). This indicates that the cell value of 786-0 cells transfected with the VHL gene is significantly reduced.

### 3.4. Detection of Transfection Efficiency by Different Transfection Methods

Liposome-mediated gene transfection is currently the most commonly used in vitro transfection method. We compared the efficiency of ultrasound microbubble-mediated gene transfection and liposome transfection. 48 hours after transfection, the transfection efficiency of pEGFP-VHL can be observed using a fluorescence microscope. Based on Figure 5, the transfection efficiency of the ultrasound microgroup (18.27% ± 2.83%) was lower than that of the liposome group (35.55% ± 2.77%). The transfection efficiency of the ultrasound microbubble group was improved within a certain range (Figure 5).

### 3.5. MTT Test on Cell Viability

We used ultrasound microbubble-mediated gene transfection and liposome transfection to transfect the empty vector into 786-0 cells. After 48 hours, the MTT experiment was used to examine the effect of two transfection methods on cell viability. Based on Figure 6, there was no significant difference in the effect of the two transfection methods on cell viability. The ultrasound microbubble group: 95.47% ± 8.04%, the liposome group: 90.63% ± 9.52%. 48 hours after transfection of 786-0 cells, the MTT experiment was used to examine the effects of the two transfection methods on cell viability. No significant difference exists between ultrasound microbubble group and the liposome group on cell viability.

## 4. Discussion

Kidney cancer is a common tumor in urology [9]. It is regrettable that about 30% of patients have reached the late stage after the diagnosis. The current treatment methods are mainly surgery plus biological therapy and radiotherapy and chemotherapy [8]. Renal cell carcinoma has poor sensitivity to radiotherapy and chemotherapy, especially for patients with advanced stage, metastasis, or recurrence. Finding a more effective treatment method has very important clinical significance for improving the treatment effect of kidney cancer [10].

Finding a more effective treatment method has very important clinical significance for improving the treatment effect of kidney cancer. Similar to other malignant tumor cells, apoptosis defects are a distinctive feature of kidney cells, showing an imbalance between proliferation and apoptosis and resistance to chemotherapy drugs [11]. It contains three exons and is located in the 3p25-26 region. Encoding product VHL protein (pVHL), pVHL includes two domains a and 0. pVHL and Elongin B-C and CUL2 proteins form a VBC (VHL·ElonginB/C-CUL2) complex. The VBC complex participates in the degradation of various proteins in the human body and belongs to the E3-ubiquitin protease system. In this system, pVHL specifically recognizes and binds substrate molecules through the 0 domain and binds to and presents substrate molecules through a domain to ElonginB/C, and VHL gene inactivation leads to the loss of these functions, which is conducive to the occurrence and development of tumors. Studies have shown that VHL gene mutations and hypermethylation are widespread in kidney cancer and are related to clinical stage, histological type, and lymph node metastasis.

70-80% of sporadic renal cell carcinomas have VHL gene inactivation [12]. Shiao [13] and other studies have shown 75 patients with renal cell carcinoma mainly clear cell carcinoma (60 cases). Using immunohistochemistry to detect the level of VHL protein, the expression level of VHL protein in 49 patients (65%) decreased significantly. Further research is needed. At present, there are few experimental studies on the VHL gene in vitro, adding tumor suppressor genes in tumor cells and analyzing the changes, which is helpful to reveal the molecular mechanism of tumor development.

Studies have found that increasing the expression of the VHL gene in tumor cells can effectively inhibit the proliferation of tumor cells and increase the sensitivity of tumor cells to radio chemotherapy [14]. We transfected the VHL gene into renal cancer cell line 786-0, using the RT-PCR method at the transcription level. At the same time, the growth activity of cells after transfection was detected by the MTT method. The selected 786-0 cell line itself is a cell line lacking the normal VHL gene, and the VHL gene is underexpressed. The results showed that after transfection, the expression level of the VHL gene in the 786-0 cell line was greatly increased at the transcription level [15]. MTT test showed that after VHL gene transfection, the growth activity of 786-0 was significantly inhibited. The apoptosis rate increased significantly. Compared with the transfected VHL gene, kidney cancer cell lines that were not transfected with the VHL gene had low expression of the VHL gene, cell growth activity was not inhibited, and cell apoptosis rate was low. This result is consistent with the results of Shiao et al.'s study on kidney cancer specimens. It further confirmed the important role of the VHL gene in the occurrence and development of human kidney cancer, and provided an experimental basis for gene therapy of kidney cancer. Seek new intervention targets and strategies for effective treatment of kidney cancer [16].

The issues caused by renal cell carcinoma are raised by more than 126% from 1950 to the present, and the annual mortality rate has increased by 37% [17]. The adverse reactions of this immunotherapy are obvious, and the effect is limited. Most kidney cancer patients overexpress VEGF, EGF, PDGF, TGF2a, and other growth factors due to VHL gene mutation and abnormal growth of tumor tissues resulting in HIF-related transcriptional activation. We activate Raf/MEK/ERK and PBK/Akt/mTOR pathways through autophosphorylation of receptor tyrosine kinases, causing uncontrolled cell division, proliferation, and transformation, stimulating neovascularization, and promoting tumor growth and metastasis [13]. The expressed growth factors and tumor-related molecular pathways can be used as targets for targeted therapy [18–20].

We applied ultrasound microbubble gene transfection technology and liposome gene transfection technology to transfect pEGFP-VHL into 786-0 cells, which we then measured the transfection rate by immunofluorescence [21]. The empty vector gene was transfected into renal cancer cell lines by the above two methods, respectively, and the effect of the two transfection methods on cell viability was detected by the MTT method [22]. The transfection efficiency of ultrasound microbubbles-mediated genes in vitro was still significantly lower than that of liposome-mediated gene transfection, but the transfection efficiency was improved to a certain extent compared with the blank control group. We prove that ultrasonic microbubble technology is safe and effective. We applied ultrasound microbubble method to transfect VHL plasmid into human kidney cancer cell lines, applied RT-PCR [10] method to detect the expression of the VHL gene, MTT to detect cell proliferation ability, and flow cytometer to detect apoptosis rate. The MTT test showed that the cell growth of the ultrasound microbubble group was significantly inhibited, the use of deep learning models is better for the research of this article [23], the flow cytometry test showed that the apoptosis rate of the ultrasound microbubble group increased [24, 25], and the experiment was repeated many times to show consistency in the results. It proves that the ultrasonic microbubbles transgene technology is stable and effective. Machine predictive control techniques [26] may be utilized in diagnosis of kidney cancer based on the biostatistics of VHL-gene transfection.

## 5. Conclusion

Ultrasound microbubbles gene transfection method can increase the transfection efficiency of the VHL gene into 786-0 cells within a certain range. Compared with liposome-mediated transfection, the two transfection methods had no significant difference in cell viability. The transfection efficiency of ultrasonic microbubbles with ultrasonic irradiation is still low, ultrasound microbubbles to promote gene transfection still have many problems, and such technique requires further research.

## Figures and Tables

**Figure 1:** RT-PCR detection of VHL gene mRNA expression in 786-0 cells based on (a) control group, (b) pcDNA3.1 (+) group, and (c) pcDNA3 1-VHL group.

**Figure 2:** 48 hours after transfection, the apoptotic rate of each group was detected using a loss cytometer. (a) Control group. (b) pcDNA3.1 (+) group. (c) pcDNA3 1-VHL group.

**Figure 3:** Apoptosis rate of each group 48 h after transfection.

**Figure 4:** MTT detects the activity changes of cells at 12 h, 24 h, 36 h, 48 h, 60 h, and 72 h after 786-0 transfection.

**Figure 5:** 48 hours after transfection, observe the distribution of GFP fluorescence in each group under a fluorescence microscope. (a) Control group. (b) Liposome group. (c) Ultrasound microbubble group.

**Figure 6:** Comparison of transfection of empty vector with ultrasonic microbubble method and liposome method.

## Data Availability

Data Availability Statement The image data used to support the findings of this study have been deposited in the cancer genome atlas (TCGA) (https://portal.gdc.cancer.gov/).
